The article "Combinatorial approach of in silico and in vitro evaluation of MLH1 variant associated with Lynch syndrome like metastatic colorectal cancer" was retracted in 2020. Reason: duplicated images.

# Combinatorial approach of *in silico* and *in vitro* evaluation of *MLH1* variant associated with Lynch syndrome like metastatic colorectal cancer

**DOI:** 10.1042/BSR20200225

**Published:** 2020-06-03

**Authors:** Komal Saleem, Tahir Zaib, Wei Ji, Chunhui Zhang, Qian Qin, Yusi Wang, Lidan Xu, Hanfei Yu, Siqi Zhu, Kexian Dong, Shuhan Si, Xueyuan Jia, Jie Wu, Songbin Fu, Wenjing Sun

**Affiliations:** 1 Laboratory of Medical Genetics, Harbin Medical University, Harbin 150081, China; 2 Key Laboratory of Preservation of Human Genetics Resources and Disease Control in China, Harbin Medical University, Ministry of Education, Harbin 150081, China; 3 Department of Gastrointestinal Medical Oncology, Harbin Medical University Cancer Hospital, Harbin 150040, China

**Keywords:** Colorectal cancer, In silico tools, In vitro analysis, Lynch syndrome, MLH1, WES

## Abstract

Colorectal cancer (CRC) is the third most developing cancer worldwide and Lynch syndrome (LS) accounts for 3–4% of CRC. Genetic alteration in any of DNA mismatch repair (MMR) gene is the major cause of LS that disrupt the normal upstream and downstream MMR events. Germline mutation of *MLH1* in heterozygous state have an increased risk for CRC. Defective MMR pathway mostly results in microsatellite instability (MSI) that occurs in high percentage of CRC associated tumors. Here, we reported a patient with LS like metastatic CRC (mCRC) associated with other related cancers. Whole exome sequencing (WES) of the proband was performed to identify potential causative gene. Genetic screening validated by Sanger sequencing identified a heterozygous missense mutation in exon 12 of *MLH1* (c.1151T>A, p.V384D). The clinical significance of identified variant was elucidated on the basis of clinicopathological data, computational predictions and various *in vitro* functional analysis. *In silico* predictions classified the variant to be deleterious and evolutionary conserved. *In vitro* functional studies revealed a significant decrease in protein expression because of stability defect leading to loss of MMR activity. Mutant residue found in MutL transducer domain of MLH1 that localized in the nucleus but translocation was not found to be significantly disturbed. In conclusion, our study give insight into reliability of combinatorial prediction approach of *in silico* and *in vitro* expression analysis. Hence, we highlighted the pathogenic correlation of *MLH1* variant with LS associated CRC as well as help in earlier diagnosis and surveillance for improved management and genetic counselling.

## Introduction

Colorectal cancer (CRC) is the third most prevalent cancer with significantly increased chances of extracolonic malignancies and variable expressivity [1–5]. One-third of the primary CRCs have the genetic background. Approximately 3–4% of CRCs are previously reported to account for Lynch syndrome (LS), also called hereditary non-polyposis CRC (HNPCC) [2,3,6]. Germline permutations accompanied with somatic inactivation that alter one of known DNA mismatch repair (MMR) genes (*MLH1, MSH2, MSH6* and *PMS2)* are the leading molecular cause of LS [7]. Most of the mutations in MMR genes associated with LS have a penetrance of approximately 80% for CRC, 60% for endometrial and approximately 20% for other cancers [1,3]. A germline mutation in *MLH1* specifically in heterozygous state have cumulative risk for developing CRC [8]. Genetic and modifier factors together cause epigenetic changes that result in variability of cancer and complete loss-of-function (LOF) mutations in MMR genes resulting in silencing of wild-type allele by mutant allele in somatic cells. Sporadic cases of LS like metastatic CRC (mCRC) mostly occurs as a result of somatic loss of wild-type allele leading to high microsatellite instability (MSI) being a major hallmark for cancer [9]. A number of different genetic variants are reported in different families with sharing of similar or variable genotype correlation for CRC. Approximately 90% of pathogenic mutations occur in either *MLH1* (50%) or *MSH2* (40%) while remaining 10% occurring in *MSH6* and *PMS2* [10].

DNA MMR system essentially play a fundamental role in identification and correction of replication errors by escaping the proofreading step of DNA replication complex and following the repair guide system by DNA polymerase and DNA ligase [2]. This rectification system being an evolutionarily conserved process improves and diminished the chances of spontaneous mutations to maintain genomic integrity [11,12]. MLH1, being a component of post-replicative DNA MMR system provide instructions for making a protein that plays a critical role in DNA repair. MLH1 protein interacts with PMS2 protein to form a dimeric complex of MutLα. MutLα then interacts and activates the activities of other protein complex of MutS (MutSα = MSH2+MSH6, MutSβ = MSH2+MSH3) to form a ternary coordinate complex which is involved in repairing errors during DNA replication. This heterodimeric coordinate complex of MutLα (MLH1+PMS2) and MutS (MutSα + MutSβ) repairs the DNA errors by replacing faulty DNA sequence with corrected DNA sequence. MutLα heterodimer is responsible for directing the downstream MMR events. Any change in upstream or downstream MMR events can cause mismatched DNA which disturbs ATPase activity and results in a distinct conformational change that is crucial for mismatch repairing [13]. Rather than clinical diagnosis likely for LS like mCRC, a confirmed genetic mutation in one of known MMR genes (*MLH1, MSH2, MSH6, PMS2* and *EPCAM)* should be present for the diagnosis of LS [14]. MSI and IHC analysis are highly sensitive molecular testing with concordant results demonstrating the abnormal expression of MMR proteins on tumor and for better evaluation followed by genetic testing [15]. Identification of pathogenic mutations allows the appropriate diagnosis, early prevention, supervision, and improved management of patients with LS [16].

Here, we reported a patient diagnosed with primary CRC associated with multiple metastatic tumors before the age of 40, fulfilling Amsterdam criteria II that one family member diagnosed with LS-associated cancer before age of 50 [17]. We identified a heterozygous variant of uncertain significance in *MLH1* and aimed to determine the pathogenicity or neutrality of variant by utilizing *in silico* predictions and comprehensive functional characterization.

## Materials and methods

### Study subject

A female patient, 41 years old, affected with primary CRC was recruited in the present study. She was diagnosed with CRC and multiple metastatic tumors possibly cancers of gastric wall, right adrenal gland, lung and intrahepatic portal lymph nodes. Clinical information and peripheral blood were obtained from the proband for further genetic analysis studies. The study was approved by Institutional Research Board of Harbin Medical University. Signed informed consent was provided by patient.

### Whole exome sequencing

Peripheral blood was collected into a qualified negative pressure vacuum EDTA anticoagulant tube. Genomic DNA extraction was performed using the DNeasy Blood & Tissue Kit (Qiagen, 69506, Dusseldorf, Germany) according to manufacturer’s protocol. In order to find the possible pathogenic variants, whole exome sequencing (WES) was performed using DNA extracted from blood of proband by Novogene Technology Limited-Liability Company (Beijing, China). Briefly, genomic DNA was fragmented to an average size of 180–280 bp and DNA libraries were produced using established Illumina paired-end protocols. The Illumina Novaseq 6000 platform (Illumina Inc., San Diego, CA, U.S.A.) was utilized for genomic DNA sequencing to generate 150-bp paired-end reads. Base calling analysis was performed with bcl2fastq software (Illumina). High-quality sequencing of data was performed using Burrows–Wheeler Aligner (BWA) [18] and all reads were aligned against reference human genome UCSC GRCh37/hg19. Duplicate reads were marked using Sambamba tools [19]. Variant calling, single-nucleotide variants (SNVs) and INDELs were identified using PINDEL (http://gmt.genome.wustl.edu/packages/pindel/) and SAMtools to generate gVCF [20,21]. The copy number variants (CNVs) from WES data were detected using SVD-ZRPKM algorithm CoNIFER (version 0.2.2) [22]. Annotation was performed using ANNOVAR [23].

### Pathogenic gene analysis

On the basis of target exome-based next-generation sequencing data, set of primers were designed for exon 12 of *MLH1* (forward: 5′-CAGACTTTGCTACCAGGAC-3′, reverse: 5′-CTGGGAGTTCAAGCATCT-3′) and polymerase chain reaction (PCR) was performed. PCR was performed in a final volume of 50 μl, using 4 μl of genomic DNA, 1.6 μl of each primer (10 pmol/l), 4 μl of dNTP, 0.4 μl of r-Taq DNA polymerase, 20 μl of 2× GC buffer and 18.4 μl of PCR water. PCR cycling condition was followed by a first denaturation step of 95°C for 10 min, subjected to 30 cycles of denaturation at 95°C for 30 s, annealing at 55°C for 30 s and extension at 72°C for 30 s. Reaction was terminated followed by a final extension at 72°C for 5 min. Mutation analysis was validated on the basis of Sanger sequencing results, and the NCBI (http://www.ncbi.nlm.nih.gov/genbank/) transcript sequence (*MLH1:* NM_000249.4) used as a reference to describe the nucleotide change.

### Plasmid and site-directed mutagenesis

The plasmid GV141 (pCMV-MCS-3FLAG-SV40-Neomycin/Amp^+^) containing full open reading frame of *MLH1* (Jikai GeneChem, Shanghai, China) was used as a template for introducing the mutant c.1151T>A, p.V384D via site-directed Fast Mutagenesis system (Trans BioNovo, Beijing, China). The entire coding sequence of wild-type and mutant *MLH1* constructs were verified by Sanger sequencing. Mutagenic primers designed according to kit protocol to generate specific mutation were forward: 5′-ATGCCCACCAGATGGATCGTACAGAT-3′ and reverse: 5′-TCCATCTGGTGGGCATAGACCTTAT-3′.

### Cell culture and transfection

Human embryonic kidney HEK-293T, HCT-116 and LOVO cells (purchased from ATCC, Manassas, VA) were cultured at 37°C in a humidified 5% CO_2_ atmosphere in Dulbecco’s modified Eagle’s medium and F12 medium supplemented with 10% FBS (Gibco, Karlsruhe, Germany). HEK-293T cells (3.5 × 10^5^/cells) were seeded on to poly-l-lysine-coated six-well plates 1 day before transfection, using JetPRIME reagent (Polyplus transfection, Illkirch, France) following manufacturer’s recommendation. Transient transfection of HCT-116 cells (MLH1-deficient) with control vector, plasmid encoding wild-type and mutant *MLH1* was performed using Lipofectamine 3000 (Invitrogen, Carlsbad, CA, U.S.A.), while LOVO cells (MLH1-proficient) were used as a positive control.

### Immunofluorescence

For immunofluorescence, HEK-293T and HCT-116 cells were seeded on glass coverslips in six-well plates for 24 h before transfection. After 48 h of transfection, cells were fixed with 4% paraformaldehyde for 20 min at room temperature and permeabilized with PBS-T (Triton X-100) for 10 min at 4°C followed by 30 min blocking with PBS-B (1% BSA). After blocking and washing steps, cells were overnight treated with anti-MLH1 antibody (1:100) (Proteintech®, Wuhan, China) at 4°C followed by incubation with anti-rabbit AlexaFluor® 488–conjugated antibody (1:1000) (Molecular Probes, Eugene, U.S.A.) for 1 h at room temperature. DAPI was used for staining nucleic acid. Glass coverslips fixed on slides and images were obtained using a Leica DM5000B laser scanning confocal microscope (Leica Microsystems, Solms, Germany).

### Western blot analysis

After 48 h of transfection, cells were lysed in ice-cold lysis buffer and protein concentration was determined by uptima bicinchoninic acid (BCA) protein assay (Applygen Technologies, Beijing, China). Lysates were separated by SDS/PAGE on 7.5% (w/v) acrylamide gel and transferred to polyvinylyidene difluoride (PVDF) membrane followed by incubation of blot with anti-MLH1 antibody at 1:1000 (Proteintech®, Wuhan, China) and anti-rabbit conjugated secondary antibody at 1:10000 (Rockland Immunochemicals, Gilbertsville, PA), respectively. Immunoblotting of β-actin with a monoclonal antibody (Invitrogen, U.K.) was also detected as a loading control. The signal was developed using the Odyssey CLx-imaging system (Li-COR, Lincoln, U.S.A.).

### Quantitative reverse transcription-PCR

Total RNA was isolated using TRIzol reagent (Invitrogen, U.K.) according to manufacturer’s protocol. RNA concentration was checked by Nanodrop-1000 spectrophotometer (Thermal Scientific, Wilmington, U.S.A.). The first-strand complementary DNAs (cDNAs) were synthesized by reverse transcription of 2 μg of total RNA using Transcriptor First-Strand cDNA Synthesis Kit (Roche Applied Science, Alameda, U.S.A.). Transcribed cDNA was used as template for quantitative reverse transcription-PCR (qRT-PCR). Using *ACTB* as a reference gene, qRT-PCR was performed in triplicate by LightCycler FastStart DNA Master SYBR Green (Roche Applied Science) and LightCycler detection system (Applied Biosystems). The primers used for qRT-PCR were: human MLH1: 5′-GCCACTGAGGTGAATTGGGACG-3′ (forward); 5′-GCCAGGCACTTCACTCTGCT-3′ (reverse); human ACTB: 5′-CAGAAGGATTCCTATGTGG-3′ (forward); 5′-CATGATCTGGGTCATCTTC-3′ (reverse). The relative quantitative expression was calculated via 2^−ΔΔ*C*_t_^ method.

### MTS proliferation assay

MTS, [3-(4,5-dimethylthiazol-2-yl)-5-(3-carboxymethoxyphenyl)-2-(4-sulfophenyl)-2H-tetrazolium] assay, a widely used approach for measuring cell viability was performed for the quantification of transiently transfected HCT-116 and LOVO cells (as positive control). The transfected cells absorbed the oxidized form of MTS reagent and intracellularly reduced by mitochondrial electron transport chain and oxidoreductases, with a compatible shift in its absorbance. Transiently transfected HCT-116 with wild-type, mutant or control vector, and LOVO cells were seeded in 96-well microliter plates. After 24 and 48 h, culture medium was replaced with 100 μl fresh medium and 20 μl of MTS (CellTitre 96^℗^ AQueous One Cell Proliferation Assay Solution, Promega, Madison, U.S.A.) and then incubated for 3 h at 37°C. After 2–3 h, absorbance was measured at 492 nm using TECAN Microplate Reader (BioTek, Winooski, U.S.A.). O.D value represents the proliferative activity and data were analyzed by GraphPad.Prism.v5.0.

### Statistical analysis

One-way analysis of variance (*ANOVA*) and Tukey’s Multiple Comparison Test were used for comparisons. *P*<0.05 was considered as statistically significant difference.

### *In silico* analysis

The frequency of variant was evaluated in 1000 Genome Project (TGP) (www.1000genomes.org), Exome Aggregation Consortium (ExAc) (http://exac.broadinstitute.org/) and gnomAD (http://gnomad.broadinstitute.org/). The variants were interpreted according to American College of Medical Genetics and Genomics (ACMG) guidelines [24]. To predict the significance and potential pathogenicity of mutant variant, various bioinformatics tools such as Mutation Taster (http://www.mutationtaster.org/), PolyPhen-2 (http://genetics.bwh.harvard.edu/pph2/), SIFT (http://sift.bii.a-star.edu.sg), PROVEAN (http://provean.jcvi.org/seq_submit.php) and MutPred2 (http://mutpred.mutdb.org/) [25] were used. Multivariate Analysis of Protein Polymorphisms–Mismatch Repair (MAPP–MMR) [26] for the accurate classification and interpretation of missense variation of *MLH1/MSH2* was also used to classify the variant to be deleterious or neutral. Three-dimensional conformation of wild-type and mutant proteins were analyzed by SWISS-MODEL (www.swissmodel.expasy.org/). Evolutionary conservation of mutation was checked by Aminode (www.aminode.org/) [27] and UCSC (http://genome.ucsc.edu/). RaptorX (raptorx.uchicago.edu/StructurePrediction/predict/) was also used to predict the secondary and tertiary structures of protein.

## Results

### Clinicopathological findings of patient diagnosed with LS

The proband was a 41-year-old female who was diagnosed with primary CRC at the age of 39 years. On the basis of clinical and pathological manifestations, primary CRC was found to be associated with metastatic tumors of other organs. Patient fulfilled the Amsterdam II criteria according to which affected individual was diagnosed before the age of 50 years. Moreover, due to ‘ONE CHILD’ policy in China, literature about the Chinese population is rare and resulting in a number of small families regarding fulfillment of other points of Amsterdam II criteria for the better diagnosis of disease. It remains contradictory whether the Amsterdam or Bethesda criteria are suitable for HNPCC screening in China. Hence, the present study is entirely a sporadic case due to unavailability of other siblings or family members.

### Mutation analysis found missense mutation MLH1:c.1151T>A in WES

WES was performed to identify pathogenic gene responsible for patient affected with CRC. Pathogenic analysis of WES data revealed total of 26517 variants including 16 pathogenic, 10 likely pathogenic, 2605 variants of uncertain significance (VUS) and 23886 benign variants. The WES data can be accessed at SRA accession: PRJNA574229 (www.ncbi.nlm.nih.gov/sra/PRJNA574229).

After comprehensive screening of pathogenic mutations in WES data, we found a heterozygous missense mutation in *MLH1* with minor allele frequency (MAF) < 0.01. Additionally, variants of other MMR genes were observed in patient’s WES data (Table 1). A heterozygous missense mutation (NM_000249.4:exon12:c.1151T>A, p.V384D) of *MLH1* detected by WES was validated by Sanger sequencing in the proband (Figure 1). Although, MLH1:c.1151T>A;p.V384D mutation has been reported and evaluated in eight different case–control studies from 1998 to 2016 (six studies in China, one in Japan and one in Korea) [28–33] listed in Supplementary Table S1. For the first time, this mutation had been reported in a study among East Asian (Chinese) patients affected with CRC but not among Europeans [34]. Functional and predictive evaluation of the identified variant was not done previously, and the variant was reported as nonfunctional polymorphism being confined only to East Asian population [34]. Though, all other previous studies show the inconclusive results. Thus, for the precise and better assessment of the possible association of the effect of this variant, two comprehensive meta-analysis studies were conducted by Chen et al. (2015) and Zare et al. (2018) [35,36] (Supplementary Table S2). A recently conducted conclusive meta-analysis study (2018) is inconsistent with previous meta-analysis in 2015. This meta-analysis gives a supportive briefing and significant association of *MLH1*:c.1151T>A variant with CRC-susceptibility in Asian population. According to meta-analysis study, this variant was associated with increased risk of CRC among Asians but not among Caucasians. This *MLH1* mutation identified in our patients was not found in the 82-control unrelated patient’s WES data.

**Figure 1:** Sanger sequencing results for verification of missense variant in exon 12 of *MLH1* (**A**) A heterozygous nucleotide change (c.1151T>A) in the patient, leading to an amino acid change from Valine (V) to Aspartate (D) at position 384 (p.V384D) and (**B**) normal reference sequence.

**Table 1:** Variants in different MMR genes found in WES data

Gene	Transcription	Genotype	Nucleotide change	Amino acid change	Mutation type	ExAC_ALL Frequency	ExAC_EAS Frequency	1000 Genome project
*MLH1*	NM_000249	Heterozygous	c.T1151A	p.V384D	Missense	0.0028	0.0385	7.7e-05
*MSH2*	NM_000251	Heterozygous	c.C1168T	p.L390F	Missense	0.0017	0.0217	-
*MSH6*	NM_000179	Heterozygous	c.A3488T	p.E1163V	Missense	0.0012	0.0138	7.7e-05
*MSH3*	NM_002439	Heterozygous	c.G169C	p.A57P	Missense	8.07e-05	0	-
*MUTYH*	NM_001048171	Heterozygous	c.1435-1G>A	-	Splicing	-	-	-

### The missense variant *MLH1:c.1151T>A* was predicted to be deleterious by computational analysis

In order to further elucidate the pathogenicity of variant, a comprehensive functional characterization accompanied with computational analysis was carried out on the basis of patient clinicopathological data.

By utilizing various prediction tools, we analyzed the variants identified in proband (Table 2). We found their population frequencies were either higher than 0.01 or they were predicted to be benign by computational analysis. Missense mutation c.1151C>T in exon 12 of *MLH1* was predicted as pathogenic by PolyPhen-2 with a score of 0.998 (Figure 2A). SIFT with a score of 0.0 and PROVEAN with a score of -5.622 (cutoff = −2.5) predicted the mutation *MLH1*:c.1151T>A to be deleterious (Figure 2B). Mutation Taster also predicted the mutation *MLH1*:c.1151T>A as disease causing with a probability value of 1 (Figure 2C). MutPred2, a predictor for inferring the molecular and phenotypic impact of amino acid variants predicts the mutation to be pathogenic with a score of 0.786. Mutpred2 predicts the molecular mechanism of mutation that it may cause altered transmembrane (*P*<0.02), loss of proteolytic cleavage at D387 (*P*<1.2e-03) and gain of sulfation at Y379 (*P*<0.03) (Figure 2D). MAPP–MMR tool interprets *MLH1:*V384D missense variant as deleterious with a score of 5.120 (Figure 2E). MAPP–MMR score for any missense variants greater than threshold score 4.5 was considered to be deleterious.

**Figure 2:** *In silico* predictions for the missense mutation *MLH1*:c.1151T>A; p.V384D (**A**) Pathogenic properties of missense variant, according to Polyphen2_HVAR. (**B**) Deleterious effect of mutant protein via PROVEAN. (**C**) Mutation taster predictions for *MLH1* variant. (**D,E**) Predictors for inferring the molecular and phenotypic impact of amino acid variants, Mutpred2 predictor score and MAPP–MMR tool prediction. (**F**) Multiple sequence alignments or evolutionary constraints regions generated by Aminode. (**G**) Swiss homology model for protein structure of wild-type and mutant MLH1 depicting the difference in size, shape and chemical structure of Valine and Aspartate.

**Table 2:** Bioinformatics prediction of mutant variants

Variants	Mutation Taster	Polyphen2_HVAR	SIFT	Mutation Assessor	PROVEAN
*MLH1*:exon12:c.T1151A:p.V384D	1, D^1^	0.998, D	0.0, D	2.745, M^4^	Del^5^
*MSH2*:exon7:c.C1168T:p.L390F	1, D	0.405, B^2^	0.009, D	2.58, M	N^6^
*MSH6*:exon6:c.A3488T:p.E1163V	1, D	0.411, B	0.016, D	2.64, M	N
*MSH3*:exon1:c.G169C:p.A57P	1, D	-	0.397, T^3^	0.345,N	N
*MUTYH*:exon15:c.1435-1G>A	1, D	-	-	-	-

Abbreviations: ^1^, Disease causing; ^2^, benign; ^3^, tolerable; ^4^, medium; ^5^, deleterious; ^6^, neutral.

Furthermore, Aminode evolutionary constrained regions (ECRs) and multiple sequence alignments of MLH1 protein showed that the mutation occurred within a highly conserved amino acid, suggesting its critical physiochemical function (Figure 2F).

A Swiss built homology model of wild-type and mutant MLH1 proteins revealed that p.V384D was located in the MutL transducer domain that affects both structure and function of the protein (Figure 2G). Wild-type residue and newly introduced mutant residue differs in size, charge and hydrophobicity value. The wild-type residue Valine (V) was neutral, smaller and more hydrophobic than negatively charged mutant residue Aspartate (D) (HOPE: http://www.cmbi.ru.nl/hope/). RaptorX also predicted that as compared with wild-type residue (Val), the mutant residue (Asp) is less buried and more exposed, which causes structural disorder of protein (Supplementary Figure S1).

Multiple programs agreed on the deleterious effect of variant showing prediction significantly related with the biological effect in cell model (Supplementary Table S3).

### The translocation and expression of MLH1 were reduced in MLH1:c.1151T>A transfected cells

MLH1 being nuclear protein is primarily localized in the nucleus. The *MLH1*:c.1151T>A mutation occurs within the highly conserved MutL transducer domain, a region that has important function in protein structure and interaction. We assumed that as a result of this mutation, protein may have altered intracellular translocation, which would prevent MLH1 from proper interaction and functioning. To check the difference between subcellular localization of wild-type and mutant protein, we performed immunofluorescence assay. After 48 h transfection, immunofluorescence in both HEK-293T and HCT-116 cells showed that MLH1-WT was completely localized into the nucleus with normal distribution. However, *MLH1*:c.1151T>A mutant showed reduced expression with slightly localized distribution, which means that cells showed equal localization in both nucleus and cytoplasm (Figure 3).

**Figure 3:** Localization of MLH1 wild-type and mutant in HEK-293T and HCT-116 cells by immunofluorescence (**A**) HEK-293T and (**B**) HCT-116 cells expressing MLH1 wild-type and mutant MLH1:c.1151T>A, were fixed with 4% paraformaldehyde and processed for immunofluorescence using anti-MLH1 antibody and anti-rabbit AlexaFluor® 488–conjugated antibody. Nuclei were stained with DAPI (in blue). Bars indicate 50 μm.

Furthermore, qRT-PCR analysis was performed with RNA isolated from the same transfected cells used for protein expression analysis. The relative mRNA values were normalized to reference ACTB. A significant decrease in MLH1 mRNA expression in MLH1:c.1151T>A cells compared with MLH1 wild-type cells was observed (Figure 4A). The expression analysis of protein extracts from transfected HEK-293T and HCT-116 cells was quantified by Western blot. Quantification results showed a significant reduction in the expression of MLH1:c.1151T>A as compared with MLH1-WT (Figure 4B,C).

**Figure 4:** Expression analysis of MLH1 wild-type and MLH1*:*c.1151T>A mutant in HEK-293T and HCT-116 cells (**A**) qRT-PCR expression analysis in HCT-116 cells. (**B**) Western blot analysis in HEK-293T cells and (**C**) HCT-116 cells. Three independent Western blot analyses effectively showed the same results. *P<0.05, ***P<0.001, by *ANOVA* and Tukey’s Multiple Comparison Test.

### The MLH1 variant could enhance cell proliferation in *in vitro* functional assay

MTS reagent, an indicator of mitochondrial activity and ATP release, was used to analyze the effect of MLH1 on cell proliferation. Proliferation of colon cancer HCT-116 cells expressing MLH1-WT was lower as compared with positive control LOVO cells, HCT-116 cells transfected with a control vector or cells expressing MLH1:c.1151T>A (Figure 5). Significant changes in proliferation of HCT-116 cells indicate that mutant MLH1 failed to regulate proliferation but show decrease in protein expression because of functional impairment and repair-deficient protein stability. It is also found that rapidity of cell proliferation depends on nucleolar size. We confirmed in our HE-staining results performed on patient dissected tissue that nucleolar size inside nucleus of cells indicates the rapid cell proliferation in tumor tissues (Supplementary Figure S2).

**Figure 5:** Proliferative activity of HCT-116 transfected cells The proliferative assay were performed with the HCT-116 cells transfected with vector control, MLH1-WT, or MLH1:c.1151T>A, and LOVO positive control cells. The proliferation activity was determined 24 and 48 h after transfection. Data shown are mean of five individual experiments. ***P<0.001 shows the significant proliferative difference between MLH1 wild-type and MLH1*:*c.1151T>A mutant.

### ACMG evaluation for MLH1 variant

ACMG guidelines were followed for evaluating the pathogenicity of the identified variant [24]. According to strong validation as a well-established *in vitro* functional studies support the damaging effect on gene or gene product (pathogenic strong (**PS3**)). One moderate validation (pathogenic moderate (**PM1**)) also supports the pathogenicity of mutant as it is located in mutational hotspot. Three supporting criteria, i.e. missense variant in a gene with low rate of benign variation and have a role in common mechanism of disease (pathogenic supporting (**PP2**)), multiple lines of computational evidences showed deleterious effect (**PP3**) and patient’s phenotype highly specific for disease with single gene etiology (**PP4**) also supports the pathogenicity of variant. On the basis of classification (Table 3), *MLH1* missense variant c.1151T>A has one strong (**PS3**), one moderate (**PM1**) and three supportive (**PP2, PP3, PP4**) evidence of pathogenicity, fulfilled the criteria of ACMG for ‘likely-pathogenic’ variant under categories two and three. Hence, *MLH1* variant is classified with an evidence of pathogenicity by (ACMG) standards and guidelines.

**Table 3:** ACMG guidelines to check the evidence of pathogenicity for MLH1:c.T1151A;V384D

ACMG priority	Items	Description
PS	PS3	Well-established *in vitro* or *in vivo* functional studies supportive of damaging effect on gene or by product
PM	PM1	Located in mutational hotspot or well-established functional domain
PP	PP2	Missense variant in a gene with low rate of benign variation and have role in common mechanism of disease
	PP3	Multiple lines of computational evidence support deleterious effect
	PP4	Patient’s phenotype or family history highly specific for disease with single gene etiology

## Discussion

In the present study, we identified and functionally characterized a heterozygous missense VUS (c.1151T>A, p.V384D) in exon 12 of *MLH1* in a Chinese patient with LS like mCRC. Based on the clinicopathological data, *in silico* predictions and expression analyses results, we validated *MLH1* variant to be likely-pathogenic. *MLH1*:c.1151T>A variant had already been reported in a study and recognized as nonfunctional polymorphism being confined only to East Asian (Chinese) population affected with CRC but not among Europeans [34]. Hence, for Chinese population (c.1151T>A) rs63750447 or ‘A’ variant allele showed increase risk for LS or CRC’s, while a protective or shielding effect among Europeans. In addition, we also identified other heterozygous missense mutations in *MSH2, MSH6* and *MSH3* genes, an interesting though rare case but on the basis of multifactorial discordant predictions. We classified variants in these genes to be non-pathogenic for this patient. Co-segregation of morbific variants with disease was an evidence to evaluate the pathogenicity of variants [13]. But our case was considered to be sporadic because of unavailability of complete family data. More than 88% of LS families have been detected with germline mutations in MMR genes following the requirements of Amsterdam criteria [37]. But it remains still contradictory whether the Amsterdam or Bethesda criteria’s are suitable for LS screening in China.

Based on the InSIGHT five-tier system [38], up till now 1344 *MLH1* variants have been registered for LS associated CRCs [39]. According to HGMD database, 1069 different types of mutations in different exons of *MLH1* has been reported (Figure 6A,B). Approximately 50% of LS like CRC cases with a known gene mutation are associated with genetic alterations in *MLH1* gene. LS increased the cumulative risk of many cancer types, predominantly cancers of colon and rectum (collectively recognized as CRC) as well as cancers of endometrium, ovaries, stomach, small intestine, liver, gallbladder duct, upper urinary tract and brain [37]. More than 33% of mutations identified in *MLH1* are missense with unknown clinical significance and recognized as VUS (Figure 6A). Some VUS have increased proficiency in mismatch repairing but show reduced expression because of decrease in protein stability. Mostly, strong pathogenic variants show decrease in protein expression and stability because of repair deficiency. It is reported that sporadic cases of CRC specifically LS occurs as a result of somatic loss of WT allele leading to high MSI and being a major hallmark for cancer [9]. Somatic mutations in MMR genes explain the absence of germline mutations and promoter methylation in half of MMR-deficient tumor cells [40,41]. Families with MMR-proficient tumors rarely have MMR gene mutations even they follow Amsterdam criteria. Because of this heterogeneity most of predisposing genetic factors and mutations remain unknown. It is found that different missense variants show heterogeneity by differently affecting the protein structure and function [42]. Moreover, a heterogeneity is also examined in tumor MSI phenotypes [43]. *MLH1* mutations being heterogenic cause different variants of LS like Turcot syndrome and Muir–Torre syndrome. Hence, it is found that *MLH1* genetic alterations are causative factors for both syndromic and non-syndromic LS.

**Figure 6:** Overview of mutation distribution per *MLH1* exons (**A**) Reported mutation types in *MLH1*. (**B**) Genomic structure and allelic spectrum of MLH1 mutations reported for LS.

Quantitative expression analysis for identified variant *MLH1*:c.1151T>A showed a significant reduction as compared with wild-type *MLH1*. It is reported that variants in certain domains of *MLH1* can severely affect the expression by destabilizing the functionality of proteins. Furthermore, proliferative activity of HCT-116 cells transfected with *MLH1* wild-type showed reduced activity compared with control plasmid or mutant *MLH1:*c.1151T>A. In the evidence of previous studies [44,45] these results revealed that mutant *MLH1* failed to regulate the proliferation and rapid proliferative activity depending on nucleolar size [46]. Various bioinformatics tools such as Mutation taster, Mutation assessor, SIFT, PolyPhen 2, PROVEAN, MutPred2 and MAPP–MMR also predicted the *MLH1* variant c.1151T>A to be pathogenic. A previous study supports the evidence of MAPP–MMR prediction by accurately predicting the damaging effect probability for validated pathogenic variants. VUS showing expression defect below than threshold value are classified as pathogenic and associated with LS [9]. It is reported that in case of *MLH1*, total MMR repair activity is compromised even if 25% of expression is lost. But on the other hand, in case of *MSH2* and *MSH6* repair activity is reduced when 75% expression is lost [43]. Recently, it is also reported that germline mutations in more than one MMR gene can more likely trigger the chances of LS. Thus, deficiency of multiple MMR genes accelerated the chances of tumorigenicity and incidence of metastatic tumors [47]. Though, in our case *MLH1* mutation was considered to be likely-pathogenic but we still believed that mutations in more than one MMR genes play a suspected role in enhancement of malignancy. Hence, further studies need to be performed in order to elucidate the origin of multiple mutations and their functional role in tumorigenicity.

It is found that *MLH1* being a nuclear protein, completely localized into the nucleus with normal distribution while mutant protein showed a little reduced expression with slightly localized distribution (Figure 3). Previously, it is reported that MLH1 variants showed three distinct translocation patterns as (i) complete nuclear localization, (ii) both nuclear (high) and cytoplasm (low) localization and (iii) equal localization in nucleus and cytoplasm. Most of the cells show nuclear localization with a combination of weak signal in cytoplasm [12]. In spite of affecting localization of protein most of missense mutations affects the stability, activity and expression of protein [9]. Recently, it is reported that nucleolus is a site of quality control for effective protein to ensure conformational maintenance. It is observed that impaired or misfolded proteins entered the nucleolus under stress conditions making the stress-sensitive nuclear proteome. Under quality control mechanism, refolding of proteins in the nucleolus during retrieval process was found to be Hsp70-dependent for localization of refolded protein. Nucleolus express chaperone like properties to promote protein maintenance under stress. But any dysfunction disrupts the quality control maintenance system of nucleolus to store misfolded proteins and lead to loss of reversibility [48]. Similarly, MMR genes being localized in nucleus has a check control system for MMRs in the DNA. Hence, any genetic alteration in one of the MMR genes might be responsible for defective MMR pathway. It is found that most of *MLH1* genetic mutations prevent the production of *MLH1* protein or lead to an altered, misfolded or nonfunctional protein that does not function properly and degraded. Thus, using pharmacological chaperones to provokes the functional rescue of misfolded protein and markedly improves the protein expression should be under consideration in future.

The strength of our study is that we used the combined approaches of *in silico* prediction tools and *in vitro* functional characterization for the evaluation of identified variant. Bioinformatics predictions were confronted and showed consistency with those of expression analysis in cell model. Our study first time predicted and confirm the pathogenicity of *MLH1*:c.1151T>A variant by emphasizing the importance of *in silico* predictions together with functional characterization. The limitation of the present study should not be ignored as we failed to check the segregation of this variant, and segregation analysis is the strong proof of any variant for confirmation. But our patient was considered to be sporadic because of the unavailability of complete family data and no family history of CRC.

## Conclusion

In conclusion, on the basis of combined approach of functional characterization and *in silico* predictions, a quantitative link between reduced expression and impaired stability of proteins among *MLH1* variant c.1151T>A, p.V384D and mCRC cancer risk was observed. Mostly, the previous studies restricted to the genetic screening and expression analysis for functional evaluation of pathogenicity. But, the main emphasis of our study focused on the combined approach of *in vitro* functional characterization and *in silico* predictions. It is concluded that diagnosis of LS cannot excluded in the presence of *MLH1* mutation in a patient with early onset CRC accompanied with associated factors. A growing number of pathogenic variations has been reported in MMR genes but most of the predisposing genetic factors and associated multiplayers behind the camera are still unknown. In future, identification and functional evaluation of MMR germline mutations needs further advancement to study their effects on subcellular localization and expression together with computational predictions for screening LS like CRCs.

## Supplementary Material

Supplementary Figures S1-S2 and Tables S1-S3

## Data Availability

The WES data can be accessed at SRA accession: PRJNA574229 (www.ncbi.nlm.nih.gov/sra/PRJNA574229. The clinical data and all the related analyzing data of the patient used to support the findings of the present study are available from the corresponding author upon request.

## Abbreviations

ACMG: American College of Medical Genetics and Genomics
ANNOVAR: ANNOtate VARiation
cDNA: complementary DNA
CRC: colorectal cancer
DAPI: 4′,6-diamidino-2-phenylindole
gVCF: genomic variant call format
HE-staining: hematoxylin staining
HGMD: human gene mutation database
HNPCC: hereditary non-polyposis CRC
Hsp70: heat shock protein70
IHC: immunohistochemistry
INDEL: insertion deletion
LS: lynch syndrome
MAPP–MMR: Multivariate Analysis of Protein Polymorphisms–Mismatch Repair
mCRC: metastatic CRC
MMR: mismatch repair
MSI: microsatellite instability
MTS: [3-(4,5-dimethylthiazol-2-yl)-5-(3-carboxymethoxyphenyl)-2-(4-sulfophenyl)-2H-tetrazolium]
PCR: polymerase chain reaction
PM: pathogenic moderate
PP: pathogenic supporting
PS: pathogenic strong
qRT-PCR: quantitative reverse transcription-PCR
VUS: variants of uncertain significance
WES: whole exome sequencing
